# Index Evaluation of Different Hospital Management Modes Based on Deep Learning Model

**DOI:** 10.1155/2022/8507288

**Published:** 2022-04-27

**Authors:** Jinai Li, Yan Wang

**Affiliations:** ^1^Jilin Medicine University Affiliated Hospital, Jilin 132013, China; ^2^The First Affiliated Hospital of Wenzhou Medical University, Wenzhou 325000, Zhejiang, China

## Abstract

In order to effectively improve the efficiency of hospital public management, we designed a hospital management index system based on deep learning model and analysed the application effect of reverse broadcast neural network model in hospital. The results show that in the performance analysis of the model, compared with other classical algorithms, the constructed model has the highest accuracy and the shortest delay. The weight analysis of each index in the model shows that the weight of rational utilization rate of beds in tertiary public hospitals is the highest, and the weight of rational utilization rate of beds in secondary public hospitals is the highest. The further analysis of the model training effect shows that the actual value of most output indexes is consistent with the predicted value, and the residual error of the predicted value is close to 0.

## 1. Introduction

In the 21^st^ century, science and technology are developing rapidly, and the era of artificial intelligence (AI) and cloud computing has come one after another. As the carrier of network interconnection, computing capabilities of computers have been improved greatly. As an emerging algorithm in recent years, deep learning is widely used in various fields such as the Internet, transportation, medical treatment, and construction. As an important part of people's lives, medical and health care has an important influence on the development and operation of this field. According to statistics, public hospitals account for more than 70% of the market share of health examination industry in 2019 in China [1]. Therefore, the effective operation and management of public hospitals is directly related to whether the residents can enjoy safe and affordable medical and health services. Therefore, application of deep learning and AI to medical and health care has become the focus of scholars in related fields to improve the operational efficiency and service quality of public hospitals.

As a pioneer who plays a basic and backbone role in China's medical service system, public hospital undertakes the main tasks of national medical and health care. In the context of medical reform, some problems in the field of health care in China have been exposed accordingly, of which the polarization of “overutilization” and “underutilization” of medical resources is more common [2, 3]. Therefore, in the new round of medical and health system reform, public hospital involves the multiple interests of different government departments, the hospital itself, medical equipment suppliers, and the majority of patients. Public hospital has become the key point of medical reform, and building an operation and management index system of public hospital based on multiple governance has become the top priority [4]. At present, there are few researches on the operation and management index system of public hospitals, and there are many ambiguities in the operation process. Studies have shown that ANN (as an algorithm of fuzzy mathematics) has a bright future in the field of fuzzy comprehensive evaluation. ANN is an information processing system that imitates the structure and function of biological neural networks. It can theoretically achieve the approximation of any function, can analyze the input and output data by setting the corresponding analysis function and parameters, and finally complete its nonlinear mapping. Thus, it has strong fault tolerance [5]. There are many studies on ANN. Mocanu et al. proposed a sparse evolutionary training algorithm for ANN, which evolved the initial sparse topology (Erdos-Renyi random graph) of two consecutive layers of neurons into a scale-free topology during the learning process and expanded the scale of ANN to the current possible level [6]. In agriculture, Caliskan et al. used ANN method to predict the chlorophyll concentration of sugar beet leaves and predicted the chlorophyll concentration by using the red, green, and blue elements in the image; and the results showed that the neural network model can better estimate the chlorophyll concentration of sugar beet leaves [7]. Hosseinzadeh et al. utilized ANN and multiple linear regression (MLR) model to evaluate the recovery efficiency of nutrients from solid waste under different earthworm compost treatments; it was found that earthworm compost significantly increased the ratio of total nitrogen (TN) and total phosphorus (TP) in the final product, and the ANN model had a better prediction effect on TN and TP [8]. For a complex organization like a public hospital, it is undoubtedly an extremely meaningful attempt to apply ANN to analyze its operation and management index system.

The contributions of this paper are as follows:

1. We have described the Internet of things technology in more detail and improved some of its functions, such as its network transmission, and we have improved its performance.
2. We applied the Internet of things to patient care in the hospital and designed a data sensitive detection based on neural network model to improve the nursing effect and work efficiency of nurses.
3. We have done many experiments to prove the superiority of the scheme based on the benchmark scheme. For example, in data collection, the performance of the scheme is improved by 2%, compared with the traditional method.

## 2. Methods

### 2.1. Public Hospital

The public hospital is usually the first comprehensive hospital established in the province. Through long-term efforts, it has become one of the key hospitals in the province. Public hospitals usually give more prominence to their role as market players. Nonprofit medical institutions such as public hospitals and public health centres can separate the ownership and management rights and separate management and supervision, so that public hospitals enjoy the status of an independent legal person and operational autonomy while fully enjoying human rights, financial rights, property rights, and decision-making rights [9, 10]. The health administration department is mainly responsible for health development planning, qualifications and access, standardization and norms, service supervision, and other industry functions, while other related parts also have to be managed and provided services according to their respective functions [11]. The common organizational framework for operation and management of a public hospital is shown in Figure 1. Clinical nursing work fails to integrate various nursing tasks such as basic care, observation of patients' conditions, medication, treatment, communication, and health guidance to provide continuous and full nursing care for patients. This paper uses the IoT technology to optimize the infusion process and achieve closed-loop management of medications and improve the efficiency and safety of infusion and medication administration by using a rational and effective outpatient and emergency infusion and medication management system. The system was built by applying wireless network, barcode technology, RFID, infrared tube sensing, and other technologies and was combined with actual nursing work to summarize application techniques and precautions. The system can improve the infusion environment, ensure the safety of patients' medication, reduce medical errors, and meet the mobile office needs of nurses and improve work efficiency.

The operation and management of public hospitals usually focus on three aspects: finance, medical efficiency, and medical quality. In terms of finance, the cost of income, medical revenue and expenditure balance, medical revenue and expenditure balance rate, and average annual business income per capita are used as budget indexes; in terms of medical efficiency, the average hospital stay of discharged patients, the average number of doctors discharged, and the average number of doctors' outpatients, and utilization rate of hospital bed are undertaken as evaluation indexes; in terms of medical quality, the rate of department director rounds, nosocomial infection rate, medical safety and hidden dangers, general medical case discussion, nursing quality, and surgical management are taken as evaluation indexes [12, 13].

At the same time, there are still some problems in the operation and management index system of public hospital. In terms of organizational structure, all aspects of operation and management are included in budget management. As a multilevel and extremely complex system, all employees are required to participate in the actual operation process, which imposes requirements on other nonfinancial personnel [14]. Therefore, during the operation of the huge public hospital system, more professionals and departments will be required to coordinate. The cooperation among departments is also extremely important, and their respective rights and responsibilities should have clear boundaries. The feasibility and practicality of some important indexes should be communicated and determined in time before setting [15, 16]. In addition, the regulatory system is not perfect, which leads to the inadequate implementation of the system at this stage, and the constraints of some clauses have not yet taken effect. Implementation has further led to a weaker control role of public hospitals in operation and management and further reduced the management authority. Therefore, using the neural network algorithm model for multiple and effective supervision of public hospitals will play a complementary role in its operation and management [17–19].

### 2.2. Artificial Neural Network

BP neural network (BPNN) mainly has two processes: forward calculation of data flow and backward propagation of error value. In the forward calculation, the neurons in each layer only affect the neurons in the next layer from input layer to hidden layer and to the output layer. If the output obtained in the output layer is not ideal, the error value is performed with backward propagation [20, 21]. Through the alternation of these two processes, the total error of the network is finally minimized, thereby completing the memory process of processing and storing the information as the optimal parameters. In the process of forward propagation, it is supposed there are *n* nodes in the input layer, *q* nodes in the hidden layer, and *m* nodes in the output layer. The weight of the input layer and the hidden layer is *v*_*ki*_, and the weight of the hidden layer and the output layer is *w*_*jk*_, as shown in Figure 2.

Figure 2 reveals that BPNN mainly completes the infinite close mapping from the *n*-dimensional space vector to the *m*-dimensional space vector, of which the transfer function of the hidden layer is defined as *f*_1_(.), and the transfer function of the output layer is defined as *f*_2_(.), which are given as follows:

(1) $$\begin{array}{c} z_{k}=f_{1}\left(\sum_{i=0}^{n}v_{ki}x_{i}\right),\;k=1,2,\cdots ,q,\\ y_{j}=f_{2}\left(\sum_{k=0}^{n}w_{jk}z_{k}\right),\;j=1,2,\cdots ,m. \end{array}$$

In the backward propagation, the number of *x*_1_, *x*_2_, ⋯, *x*_*p*_ input learning samples is set to *P*, and *y*_*j*_^*p*^(*j*=1,2, ⋯, *m*) can be obtained after inputting it into the network. The error function adopts the square type, and the error result of the *p*^*th*^ sample can be obtained as *Ep*:

(2) $$\begin{array}{c} E_{P}=\frac{1}{2}\sum_{j=1}^{m}{\left(t_{j}^{p}-y_{j}^{p}\right)}^{2}. \end{array}$$

In the above equation, *t*_*j*_^*p*^ refers to the expected output. For the total number of samples *P*, the global total error is given as follows:

(3) $$\begin{array}{c} E=\frac{1}{2}\sum_{p=1}^{P}\sum_{j=1}^{m}\left(t_{j}^{p}-y_{j}^{p}\right)=\sum_{p=1}^{P}E_{P}. \end{array}$$

Secondly, the weight value of the output layer changes, *w*_*jk*_ is adjusted with cumulative error BP algorithm, so that the global total error *E* can be reduced gradually, as shown in the following equation:

(4) $$\begin{array}{c} \Delta w_{jk}=-\eta \frac{\partial E}{\partial w_{jk}}=-\eta \frac{\partial }{\partial w_{jk}}\left(\sum_{p=1}^{P}E_{P}\right)=\sum_{p=1}^{P}\left(-\eta \frac{\partial E_{P}}{\partial w_{jk}}\right). \end{array}$$

In equation (4), *η* refers to the learning rate. The error signal can be defined as the following equation:

(5) $$\begin{array}{c} \delta_{yj}=\frac{\partial E_{p}}{\partial S_{j}}=\frac{\partial E_{p}}{\partial y_{j}}\cdot \frac{\partial y_{j}}{\partial S_{j}}. \end{array}$$

It can be written as (6) based on the chain theorem.

(6) $$\begin{array}{c} \frac{\partial E_{p}}{\partial S_{j}}=\frac{\partial E_{p}}{\partial y_{j}}\cdot \frac{\partial y_{j}}{\partial S_{j}}=-\delta_{yj}z_{k}=-\sum_{j=1}^{m}\left(t_{j}^{p}-y_{j}^{p}\right)f_{2}^{\prime }\left(S_{j}\right)z_{k}. \end{array}$$

Thus, the final weight value of each neuron in the output layer can be adjusted into

(7) $$\begin{array}{c} \Delta w_{jk}=\sum_{p=1}^{P}\sum_{j=1}^{m}\left(t_{j}^{p}-y_{j}^{p}\right)f_{2}^{\prime }\left(S_{j}\right)z_{k}. \end{array}$$

Finally, the weight value of the hidden layer changes, which is similar to the weight value of the output layer, and the equation can be obtained as follows:

(8) $$\begin{array}{c} \Delta v_{ki}=\sum_{p=1}^{P}\sum_{j=1}^{m}\eta \left(t_{j}^{p}-y_{j}^{p}\right)f_{2}^{\prime }\left(S_{j}\right)w_{jk}f_{1}^{\prime }\left(S_{k}\right)x_{i}. \end{array}$$

In actual network design, the number of hidden layer nodes is usually determined according to the complexity of the actual issue, and the principle is more nodes after less nodes. In real life, most data are nonlinear and separable, and the activation function is to introduce some nonlinear factors so that the neural network can solve more complex issues. The activation function has the characteristics of nonlinearity, differentiability, and monotonicity. Common activation functions include sigmoid function, tanh function, and elu function [22]. The expression of the sigmoid activation function is given as follows:

(9) $$\begin{array}{c} f\left(x\right)=\frac{1}{1+e^{-x}}. \end{array}$$

The value range of this function is (0, 1), and it has the property of continuous smoothness and is easy to derive. Compared with the sigmoid activation function, tanh function is more widely used, and it can be expressed as follows:

(10) $$\begin{array}{c} f\left(x\right)=\frac{1-e^{-2x}}{1+e^{-2x}}. \end{array}$$

The value range of this function is (−1, 1), and it is also called the hyperbolic tangent function. The ReLu function has a faster convergence speed in the optimization algorithm and can be implemented faster when it involves exponential operations. It is defined as follows:

(11) $$\begin{array}{c} f\left(x\right)=\max\left(0,1\right). \end{array}$$

This function effectively alleviates the gradient disappearance, making its derivative value 0 or 1, and it provides the neural network with sparse expression capabilities [23].

### 2.3. Construction for Operation and Management Model of Public Hospital Based on Artificial Neural Network

In this article, the existing operation and supervision models of public hospitals in China and the commonly used supervision indexes and their formulation methods are investigated through literature research and typical survey methods. At the same time, the supervision effect and the problems and deficiencies in the index system are investigated and analysed. On this basis, the public hospital regulatory indexes based on multiple supervision are formulated in line with the principles of simplicity, efficiency, and feasibility. Therefore, a three-layer BPANN is established, with operation management indexes of public hospital as the input layer nodes, comprehensive operation relative efficiency of public hospital as the output layer node, and 4 as hidden layer nodes, as shown in Figure 3.

In the above research model, the selected operation and management materials are mainly based on the public welfare and efficiency of public hospitals, which mainly include 5 secondary indexes and 7 tertiary indexes. In addition, the interests of multiple parties are reflected, as shown in Table 1.

In order to eliminate the influence of the difference in different indexes on the accuracy of the network, the indexes are optimized, including the proportion of medical revenue to business revenue, the nondebt ratio, the proportion of nurses to the total number of doctors and nurses, the proportion of salary and welfare expenditure to total expenditure, and the reasonable utilization rate of beds, normalized total asset return rate, and the proportion of income to total income and expenditure. In the model, the data of input sample public hospitals (120, obtained through on-site research and related information) is adopted to train the network model until the error meets the requirements, and the weight matrix *W* from the input layer to the hidden layer and the weight matrix *V* from the hidden layer to the output are obtained. In addition, weights of all nodes in the input layer (i.e., 7 supervision indexes) are calculated by using W and V.

### 2.4. Simulation Experiment

The MATLAB simulation platform is adopted to simulate and analyze the model, and the proposed model algorithm BPANN is compared with other classic algorithms for evaluation to ensure the objectivity of the experiment. Other classic algorithms include convolutional neural network (CNN), Google inception net (GoogLeNet), visual geometry group 16 (VGG16), residual network (ResNet), and multilayer perceptron (MLP). The weight value of each index and the model training effect are analysed further with statistical methods [24, 25]. The hardware used in this experiment is a Lenovo Y500 notebook, the CPU model is i5-3210m, and the memory is 8 GB. The software platform is Python 3.5.3, which mainly uses three libraries: pandas, NumPy and Sklearn. The hyperparameter is set to batch size of 128 and the learning rate is 0.001. Adam optimizer is used.

## 3. Results

### 3.1. Comparison on Performances of Various Algorithm Models

The constructed model is compared with CNN, GoogLeNet, VGG16, ResNet, and MLP algorithms to judge its accuracy and operating efficiency, and the results are shown in Figures 4 and 5.

Through the comparison and analysis of the accuracies of various algorithm models are given in Figure 4, it reveals that accuracy of the constructed model is the highest, followed by the VGG16, while the accuracies of the other algorithms are not different from each other obviously. Therefore, the performance of the proposed algorithm model in the operation and management index system of public hospital is significantly better than other algorithms.

Figure 5 shows the comparison and analysis of the time delays of multiple algorithm models, and it reveals that the established BPNN has the shortest time delay. When the number of iterations is 100, the time delay is less than 20 ms, so its operating efficiency is the highest.

### 3.2. Weight Results for Indexes of Neural Network Models

The operating indexes of public hospital in the neural network model are analysed, and the weights obtained are shown in Figure 6. It discloses that in the tertiary public hospital, the reasonable utilization rate of beds has the highest weight, while the normalized total asset return rate is the smallest, which is less than 5%; in the second-level public hospital, the normalized total asset return rate is the highest (0.342), and the proportion of income to total income and expenditure has the smallest weight, which is 0.22.

### 3.3. Training Results of Neural Network Model

The training results of the neural network model can be used for in-depth evaluation, as shown in Figures 7 and 8.

Figures 7 and 8 indicate that in the training and analysis of the tertiary and the second-level public hospital, the actual values of most output indexes are consistent with the predicted values, and the residuals of most of the predicted values are around 0. Therefore, the training error of the neural network model is small, so it has certain reliability[26, 27].

## 4. Conclusion

With the rapid development of technology, deep learning algorithms are more and more widely used, but their performances have to be improved further in real life. The deep learning algorithms are applied to the operation and management index system of public hospital, and an ANN-based operation and management model of public hospital is constructed and performed with simulation and statistical analysis. The results disclose that the established model has high accuracy, low time delay, clear weight of each index, and actual values of most output indexes matching to the predicted values, so it can provide experimental basis for operation and management index system of public hospitals in future. However, there are still some shortcomings in this article. For example, the sample size is small due to limited time and energy. Therefore, in the follow-up research, the sample size should be further expanded so that the accuracy of the weight of each index can be improved and representative, and the operation and management of the public hospital in the later period can be more standardized and clearer.

## Figures and Tables

**Figure 1:** Schematic diagram for organizational framework of operation and management of a public hospital.

**Figure 2:** Topological graph of BPNN with three layers.

**Figure 3:** Flowchart for operation and management model of public hospital based on artificial neural network.

**Figure 4:** Comparison on accuracies of various algorithm models.

**Figure 5:** Comparison on time delays of various algorithm models.

**Figure 6:** The weight of each index in the operation management model of public hospital based on ANN: (a) the proportion of medical revenue to business revenue; (b) the nondebt ratio; (c) the proportion of nurses to the total number of doctors and nurses; (d) proportion of salary and welfare expenditure to total expenditure; (e) reasonable utilization rate of beds; (f) normalized total asset return rate; (g) proportion of income to total income and expenditure.

**Figure 7:** Related training results of the tertiary hospital: (a) the measured value and predicted value of relative efficiency; (b) the predicted value and residual error of relative efficiency.

**Figure 8:** Related training results of the secondary hospital: (a) the measured value and predicted value of relative efficiency; (b) the predicted value and residual error of relative efficiency.

**Table 1:** Initial screening for operation and management indexes of public hospital.

Secondary index	Tertiary index	Principle stockholders
Economic operation	Proportion of medical revenue to business revenue	Price department
	Nondebt ratio	State-Owned Assets Supervision and Administration Commission
Service quality	Proportion of nurses to the total number of doctors and nurses	Patients
Staff welfare	Proportion of salary and welfare expenditure to total expenditure	Medical staff
Work efficiency	Reasonable utilization rate of beds	Health administration
Management efficiency	Normalized total asset return rate	State-Owned Assets Supervision and Administration Commission
	Proportion of income to total income and expenditure	Hospital

## Data Availability

The datasets used in this paper are available from the corresponding author upon request.
